# Transcriptional repression of SOCS3 mediated by IL-6/STAT3 signaling via DNMT1 promotes pancreatic cancer growth and metastasis

This article has been retracted.

**DOI:** 10.1186/s13046-016-0301-7

**Published:** 2016-02-04

**Authors:** Li Huang, Bin Hu, Jianbo Ni, Jianghong Wu, Weiliang Jiang, Congying Chen, Lijuan Yang, Yue Zeng, Rong Wan, Guoyong Hu, Xingpeng Wang

**Affiliations:** Department of Gastroenterology, Shanghai General Hospital, Shanghai Jiaotong University School of Medicine, 100 Haining Road, Shanghai, Hongkou District 200080 China

**Keywords:** Interleukin-6, Signal transducer and activator of transcription 3, Suppressor of cytokine signaling 3, DNA Methyltransferase 1, Methylation, Pancreatic ductal adenocarcinoma

## Abstract

**Background:**

Previous studies have investigated the sustained aberrantly activated Interleukin-6 (IL-6)/signal transducer and activator of transcription 3 (STAT3) signaling pathway is crucial for pancreatic cancer growth and metastasis. Suppressor of cytokine signaling 3 (SOCS3), as a key negative feedback regulator of this signaling pathway, is usually down-regulated in various cancers. In the present study, we aim at exploring the biological function and the underlying molecular regulation mechanisms of SOCS3 in pancreatic cancer.

**Methods:**

The expression of SOCS3 and other genes in pancreatic cancer was examined by Quantitative real-time PCR, western blotting and immunohistochemical staining. The interaction between pSTAT3 and DNA Methyltransferase 1 (DNMT1) was investigated by co-immunoprecipitation assay. Luciferase reporter assay was used to investigate the transcriptional regulation of pSTAT3 and DNMT1 on the SOCS3 gene. The effects of SOCS3 on the biological behavior of pancreatic cancer cells were assessed both in vitro and vivo. Furthermore, we performed a comprehensive analysis of the expression of SOCS3 in a pancreatic cancer tissue microarray (TMA) and correlated our findings with pathological parameters and outcomes of the patients.

**Results:**

We showed that SOCS3 expression was decreased in phosphorylated STAT3 (pSTAT3)-positive tumors and was negatively correlated with pSTAT3 in pancreatic cancer cells. We also found that IL-6/STAT3 promoted SOCS3 promoter hypermethylation by increasing DNMT1 activity; silencing DNMT1 or 5-aza-2-deoxycytidine (5-AZA) treatment could reverse the down-regulation of SOCS3 mediated by IL-6. Using co-immunoprecipitation and luciferase reporter assays, we found that STAT3 recruited DNMT1 to the promoter region of SOCS3 and inhibited its transcriptional activity. Overexpression of SOCS3 significantly inhibited cell proliferation, which may be due to the increase in G1-S phase arrest; overexpression of SOCS3 also inhibited cell migration and invasion as well as tumorigenicity in nude mice. Pancreatic cancer tissue microarray analysis showed that high SOCS3 expression was a good prognostic factor and negatively correlated with tumor volume and metastasis.

**Conclusion:**

We demonstrated that activated IL-6/STAT3 signaling could induce SOCS3 methylation via DNMT1, which led to pancreatic cancer growth and metastasis. These data also provided a mechanistic link between sustained aberrantly activated IL-6/STAT3 signaling and SOCS3 down-regulation in pancreatic cancer. Thus, inhibitors of STAT3 or DNMT1 may become novel strategies for treating pancreatic cancer.

**Electronic supplementary material:**

The online version of this article (doi:10.1186/s13046-016-0301-7) contains supplementary material, which is available to authorized users.

## Background

Pancreatic ductal adenocarcinoma (PDAC) is currently one of the deadliest solid tumors, with a median survival duration of approximately 6 months following diagnosis and a five-year survival rate of less than 5 % [1]. PDAC has very few early symptoms and develops rapidly; thus, most carcinomas are confirmed in an advanced stage and are not treatable by surgery [2]. The dense desmoplastic stroma of PDAC contains activated fibroblasts, inflammatory cells, various inflammatory cytokines and growth factors that lead to an inflammatory microenvironment that provides survival and proliferative signals to promote tumor initiation, progression and treatment resistance [3, 4]. Thus, despite exciting recent progress in biological target therapy for tumors, most targeted therapies show no clinical benefit in PDAC [5].

Chronic inflammation is an important risk factor for cancer development at many sites [6]. The inflammatory microenvironment exposures induce epigenetic modifications by DNMTs, altering the expression of tumor suppressor genes, which promotes PDAC tumorigenesis and progression [7, 8]. As an important member of the tumor inflammatory microenvironment, the pro-inflammatory cytokine IL-6 is involved in pancreatic cancer development [9, 10] and directly affects cancer cell growth and survival through activation of STAT3 [11–13]. The activated pSTAT3 functions as nuclear transcription factor regulating genes involved in tumor proliferation, survival, angiogenesis and invasion [14]. SOCS family is cytokine-inducible negative regulators of this cytokine signaling. As a member of the family, SOCS3 can be induced by IL-6/STAT3 signal axis and plays an important role in preventing excessive activation of the signaling pathway. SOCS3 blocks the phosphorylation of STAT3 by inhibiting Jak-2 directly [15]. The function of SOCS3 in cancer remains controversial as SOCS3 has been shown to possess both tumor limiting and tumor promoting properties. SOCS3 was reported to function as a tumor suppressor in breast cancer [16], hepatocellular cancer [17], small cell lung cancer [18], prostate cancer [19] and so on. However, other studies demonstrated that it enhanced tumor aggressiveness and associated with poor outcomes in renal cell carcinoma [20], T-cell lymphoma [21]. Few studies are available on evaluating SOCS3 expression in association to tumor biological behavior and prognosis specifically in PDAC. The aim of this study is to explore the potential roles of SOCS3 in PDAC.

The epigenetic gene silencing of SOCS3 due to promoter methylation is observed in many malignancies, including head-neck cancer [22], cervical cancer [23], pancreatic cancer [24] and hepatocellular cancer [24]. Multiple studies have demonstrated that IL-6 could promote tumourigenesis and progression by activating DNMT1, inducing aberrant DNA methylation of tumor suppressor genes and silencing their expression [24–26]. Moreover, previous studies have suggested that the IL-6/STAT3 signaling pathway is aberrantly activated in pancreatic cancer and the molecular mechanism remains unknown [27]. We thus hypothesized that the expression of SOCS3 was epigenetically silenced in pancreatic cancers owing to IL-6 induced DNMT1 expression.

In this study, for the first time, we demonstrate that activated IL-6/STAT3 signaling induced SOCS3 methylation via DNMT1, which may promote pancreatic cancer growth and metastasis both in vitro and vivo. We also provide a mechanistic link between sustained aberrantly activated IL-6/STAT3 signaling and SOCS3 down-regulation in pancreatic cancer.

## Methods

### Tissue samples, cell lines and reagents

Five pairs of primary pancreatic cancer and pericancerous tissues were obtained from Shanghai First People’s Hospital. All participants provided informed consent according to the Helsinki Declaration, and the protocol for the present study was approved by the Ethics Committee of Shanghai First People’s Hospital (Shanghai, China). The tissues were frozen at −80°C until use or fixed in formalin. Nine pancreatic cancer cell lines, Aspc1, Bxpc3, Capan1, Capan2, Cfpac, Hpaf, Panc1, Sw1990, Hs766T were cultured in RPMI 1640 or DMEM supplemented with 10 % fetal bovine serum. Human recombinant IL-6 and STAT3 inhibitor S31-201 were purchased from Sino Biological Inc. (Beijing, China) and Selleckchem (Houston, Texas, USA), respectively. 5-AZA was purchased from Sigma (St. Louis, MO, USA).

### Immunohistochemistry

Sections of 5μm from formalin-fixed and paraffin-embedded specimens were deparaffinized using xylene and rehydrated in graded ethanol. Samples were then preincubated with 3 % H2O2 to inhibit endogenous peroxides activity. Sections were incubated at 4°C overnight with primary antibodies against pSTAT3(1:100; CST), DNMT1(1:100; CST), DNMT3a(1:100; Santa Cruz), IL-6(1:50; Santa Cruz), SOCS3(1:50; Santa Cruz), and then with HRP-labeled secondary antibodies (MaxVision, China) at room temperature for 15 min, and freshly prepared 3,3′-diaminobenzidine (DAB) for color development for 5 min. In the controls, the primary antibody was replaced with phosphate-buffered saline. The evaluation of the immunohistochemical staining was performed independently by two authors without knowledge of the clinicpothological information. The intensity of immunostaining (0 = negative, 1 = weak, 2 = moderate, and 3 = intense) and the percentage of positive cells (0 % = negative, 1 %–25 %–1, 26 %–50 %–2, 51 %–75 % = 3, ≥76 % = 4) were assessed. The two scores were multiplied to give a final score and the immunohistochemical stainings were finally determined as negative: score 0; low expression: score ≤4; moderate expression: score 5–8; high expression: score 9–12.

### Protein extraction and Western blot analyses

Cells were lysed in a buffer solution containing 2 × SDS, 1 % phosphatase inhibitor and 1 % protease inhibitor. The protein concentration of the cell lysates was measured using the Pierce BCA Protein Assay Kit. Approximately 30 μg of protein from each sample was separated on 8 %–12 % SDS-PAGE and transferred to a PVDF membrane. The membrane was incubated in blocking buffer for 1 h at room temperature. The blocking buffer consisted of 5 % non-fat dry milk in Tris buffered saline containing 0.1 % Tween 20 (TBST). After washing the membrane with TBST, the membrane was incubated with pSTAT3(1:2000; CST), STAT3(1:1000;CST), DNMT1(1:1000;CST), ACTIN(1:1000;CST), DNMT3a(1:1000;CST), SOCS3(1:500;CST), CYCLIND1(1:1000;CST), BCL-2(1:1000;CST), MMP-2(1:1000;CST), MMP-9 (1:1000;CST) overnight at 4°C. Then, the membrane was washed with TBST, and incubated with secondary antibodies diluted at 1:2000 for 1 h at room temperature. The immuno-reactive protein bands were visualized using an ECL kit. Immuno-reactive band intensities were quantified using Image J software.

### Quantitative reverse transcription-polymerase chain reaction (qRT-PCR)

Total mRNA was extracted from pancreatic cancer cell lines using TRIzol reagent. Then, CDNA was synthesized from 1 μg of total RNA using oligo dT and Quant Reverse Transcriptase (Tiangen, China). Real-time quantitative PCR was then conducted using SYBR Green (Roche) according to the manufacturer’s instructions. The primers used for SOCS3 and β-ACTIN are listed in Table 1. PCR conditions were as follows: 94°C for 30 s, 60°C for 30 s and 72°C for 90 s, for 30 cycles, and a final extension at 72°C for 5 min. Relative expression levels of the genes were calculated using the 2^-ΔΔCT^ method.

**Table 1:** PCR primers

Gene	Sequence (5′-3′)	Experimental use
SOCS3	CAGCTCCAAGAGCGAGTACCA (forward)	Real-time PCR
	AGAAGCCGCTCTCCTGCAG (reverse)	
β-ACTIN	GCACCACACCTTCTACAATGAGC (forward)	Real-time PCR
	TAGCACAGCCTGGATAGCAACG (reverse)	
SOCS3(M)	TGATTAAATATTATAAGAAGGTCGGTCG (forward)	Methylation-specific PCR
	ACTAACTACGTACGAAACCGAAACG (reverse)	
SOCS3(U)	GTAGTGATTAAATATTATAAGAAGGTTGGTTG (forward)	Methylation-specific PCR
	CTAACTACATACAAAACCAAAACAA (reverse)	
SOCS3 siRNA-1	CCAAGAACCUGCGCAUCCAdTdT	RNA interference
SOCS3 siRNA-2	GGACCAAGAACCUACGCAUdTdT	RNA interference
SOCS3 siRNA-3	CCAAGAGAGCUUACUACAUdTdT	RNA interference
SOCS3 siRNA-NC	UUCUCCGAACGUGUCACGUTT	RNA interference

### Cell transfection

Lentiviral pGMLV-SC6 RNAi vectors expressing short hairpin RNA against human DNMT1 and GFP used as a negative control were constructed. High-titer lentiviral vector stock was produced in 293T cells using HG transgene reagent-mediated cotransfection with pGMLV and pUC19 packaging vectors. Freshly prepared viruses were used to infect Bxpc3 cells with rich DNMT1 expression and selected, maintained with 0.8 μg/ml puromycin. DNMT1 expression vector or the corresponding empty vector (Sino Biological Inc., China) were transiently transfected into pancreatic cancer cells using X-tremeGENE HP DNA Transfection Reagent (Roche, China).

Human SOCS3-specific short interfering RNA (siRNA) sequence and nonsense siRNA used as negative control (NC) were synthesized (Genepharma, Shanghai, China) (Table 1). Panc1 cells (2 × 10^5^) were seeded into 6-well plates and were grown until 60 %–80 % confluent. The cells were transiently transfected with 20 nmol/L of SOCS3 siRNA or NC siRNA using X-tremeGENE siRNA Transfection Reagent (Roche, China) according to the manufacturer’s instruction. After 48h, protein expression levels of SOCS3 were detected using Western blotting. The SOCS3 coding sequences were amplified and cloned into PGMLV-PA6 constructs; then, according to the manufacturer’s instructions, the lentiviral expression constructs and a packaging plasmid mix were co-transfected into HEK-293 T cells, viral particles were collected and titers were determined. Finally, Bxpc3 cells were transfected with the lentiviruses using Lipofectamine 2000.

### Methylation-specific PCR

The methylation status of the SOCS3 promoter region near the recognized STAT3-SOCS3 binding sites (−1046 through −1038, TTCCAGGAA, the start codon ATG as +1) [28–30] was determined by methylation-specific PCR (MSP) using bisulfite-modified DNA. The sequences of the methylated and unmethylated primer pairs are listed in Table 1 (methylated products: −1079 through −925, 155bp; unmethylated products: −1083 through −926, 158bp). DNA was modified using an EZ DNA Methylation-Gold^TM^ kit (ZYMO RESEARCH CORP). Amplification was achieved in a 25μl reaction volume containing 0.5μl of each primer, 2μl of modified DNA, 12.5μl 2 × Tag Enzyme (DBI, China). The PCR reaction conditions were as follows: heating at 95°C for 10 min, 35 cycles consisted of denaturation at 94°C for 15 s, annealing at 55°C for 30 s, extension at 72°C for 30 s, then a final 10-min extension at 72°C. The PCR products were visualized on a 2 % agarose gel using DuRed and UV illumination. Sss-I methylase-treated DNA (Qiagen) and unmethylated and bisulfite converted human control DNA were used as positive and negative controls, respectively.

### Co-immunoprecipitation

Total protein of cells in a 10 cm dish was lysed in 1 ml ice cold lysis buffer (RIPA). Equal aliquots (approximately 0.475 ml of each) were incubated at 4°C overnight with either 1μg rabbit anti-pSTAT3 (CST) or 1μg purified rabbit IgG (Sigma) as a control, then added to 30μl of Protein A + G Agarose (Pierce) shaken at 4°C for 4 h, and then centrifuged at 2500 g for 5 min, carefully sucked out supernatant. The precipitation was washed five times with lysis buffer, re-suspended in SDS buffer, and primary antibodies against pSTAT3 and DNMT1 were used for western blot analyses.

### Luciferase reporter assay

The human SOCS3 promoter region (−1084 through +1) including the STAT3-SOCS3 binding sites was amplified using PCR and inserted into pGL3 vector (Promega). The PCR primers were as follows: 5′ CCTTAAGCTAGC AGTAGTGACTAAACATTACA 3′ (forward, NheI), 5′ CCTTAAAGATCT GGCGCACGGAGCCAGC 3′ (reverse, BgIII) [31]. Panc1 cells (5 × 10^4^) were seeded on 24-well plates 1 day before transfection. The cells were transfected with 0.45μg reporter plasmid (pGL3-SOCS3) or DNMT1 plasmid at the same time using Lipofectamine 2000 transfection reagent. 0.05μg Renilla luciferase plasmid phRL-tk was co-transfected to normalize the transfection efficiency. Then, 24 h after the transfection, the cells were treated with 100 ng/ml IL-6 or 5μmol/L 5-AZA. Luciferase activity was measured 48 h after treatment using the Dual Luciferase Reporter Assay System (Promega). All of the assays were performed in triplicate.

### Flow cytometry

Pancreatic cancer cells that had been overexpressed or siRNA knocked down SOCS3 were trypsinized, washed in phosphate-buffered saline, and fixed in ice-cold 70 % ethanol-phosphate-buffered saline. After washing out ethanol, the fixed cells were treated with 0.01 % RNase for 10 min at 37°C and then stained with 0.05 % propidium iodide for 20 min at 4°C in the dark. The cell cycle distribution was determined using FACScan flow cytometry. Cell apoptosis and necrosis were assessed using the Annexin V-FITC apoptosis kit according to the manufacturer’s instructions.

### Cell proliferation assay

The SOCS3 gene stably transfected Bxpc3 cells (1.0 × 10^3^/well) were plated in 96-well plates (three wells per group) before measurement. Cell proliferation was analyzed using the CCK8 Cell Proliferation Assay Kit (Invitrogen, Carlsbad, California, USA). 10 μL of CCK8 was added to each well and incubated for 2 h. The number of viable cells was calculated by absorbance measurements at 450 nm.

### Wound healing assay

Cell migration was assessed using classical wound healing assays. Pancreatic cancer cells were seeded in six-well plates and transfected when they were attached. After transfection for 48 h, wounds were scratched on the monolayer of cells using 20μl pipette tips and washed twice to remove non-adherent cells. The images (100×) of the same areas were recorded using a photomicroscope at 0 h, 8 h and 24 h.

### Transwell invasion assay

For the invasion assay, the upper chamber was precoated with Matrigel (BD Bioscience) according to the manufacturer's protocols. Then, 48 h after transfection, the cells were harvested, counted and suspended in serum-free RPMI-1640 medium. Then, 1 × 10^5^ Panc1 cells or Bxpc3 cells in 100μl medium were added to the upper chamber. Medium containing 10 % FBS was added to the lower chamber as a chemoattractant. After 24h incubation, chambers were fixed with 4 % paraformaldehyde for 20 min, then 0.1 % crystal violet solution for 15 min, and then immersed in PBS for 20 min. Finally, cells in the lower chamber were counted under an inverted microscope. The cell numbers in 5 random fields of view were counted (100×).

### Tissue microarrays

A pancreatic cancer tissue microarray purchased from Xin Chao (Shang Hai) was used for immunohistochemistry analysis of SOCS3 expression. Pancreatic cancer and matched pericancerous samples were collected between 2004 and 2009 from 90 patients with informed consent. Ethical approval for the study was obtained from the ethical committee of biobank centre-associated hospitals. Clinicopathological characteristics of the tissue microarray include age, gender, tumor volume, survival time, pT, pN and pTNM classification. The information is listed in Table 2.

**Table 2:** Association between SOCS3 expression and clinicopathological parameters in pancreatic cancers

Parameter	No. of cases	Negative	Weak	Moderate	Mean Rank	*p* value
Gender						0.425
Male	57	24	27	6	44.03	
Female	33	9	23	1	48.05	
Age						0.289
< 60	41	17	22	2	42.68	
≥ 60	49	16	28	5	47.86	
Tumor Volume(cm3)						0.037
≤ 50	57	16	36	5	49.35	
> 50	33	17	14	2	38.85	
pT stage						0.584
T1	5	1	3	1	55.9	
T2	70	25	42	3	44.9	
T3	15	7	5	3	44.83	
pN stage						0.038
N0	51	14	32	5	49.9	
N1	39	19	18	2	39.74	
pTNM stage						0.001
I	40	6	29	5	55.84	
IIA	9	5	3	1	38.61	
IIB	41	22	18	1	36.93	

### In vivo tumorigenicity

All protocols for the animal studies were approved by the institutional Animal Research Ethics Board. SOCS3 overexpressed Bxpc3 cells and controls (1 × 10^7^ cells in 0.2 ml phosphate-buffered saline) were subcutaneously injected into the dorsal flank of 5-week-old nude mice; each group included 5 mice. Six weeks after injection of the cells, mice were sacrificed and the volume and weight of the tumors were recorded. The tumor volume was determined using the following formula: tumor volume (mm^3^) = length (mm) × width (mm) ^2^/2.

### Statistical analysis

The data are presented as the means ± standard deviation (SD). Quantitative RT-PCR, CCK-8 assay, cell apoptosis and cell cycle analysis, migration and invasion assay, luciferase reporter assay and nude mice tumor formation assay were assessed using one-way analysis of variance (ANOVA) for factorial design. The association between SOCS3 IHC expression and clinicopathological parameters in pancreatic cancers was analysed using Kruskal-Wallis rank sum test. The postoperative survival rate was analyzed with Kaplan–Meier method and the survival differences of patient subgroups were compared by the log-rank test. Independent variables with a *P* value <0.05 in the univariate analysis were entered into the multivariate Cox regression model. *P*–values < 0.05 were considered statistically significant, and *P*–values < 0.01 were considered highly statistically significant.

## Results

### Expression of pSTAT3 and SOCS3 in PDAC and matched pericancerous tissue

IL-6, pSTAT3, DNMT1, DNMT3a, and SOCS3 were evaluated by immunohistochemistry in five pairs of PDAC and pericancerous tissue. We showed the representative images of one pair in Fig. 1a. Immunoreactivity of pSTAT3 and DNMT1 was observed mainly in the cell nuclei, whereas IL-6, DNMT3a and SOCS3 were located mainly in the cytoplasm. Statistical analysis of the IHC scores for the specimens demonstrated that expression of IL-6, pSTAT3 and DNMT1 was significantly increased in tumor tissues, while SOCS3 expression was decreased as compared to pericancerous tissues (Fig. 1b). These data might suggest IL-6, pSTAT3, DNMT1 as oncogene and SOCS3 as tumor-suppressor gene in PDAC. Protein expression levels of pSTAT3, STAT3 and SOCS3 were also examined in the five pairs of PDACs and their matched pericancerous tissues using western blots. We found that STAT3 was obviously activated in tumor tissues, while SOCS3 protein expression was higher in their matched noncancerous tissues (Fig. 1c, Additional file 1: Figure S1A). To further determine the relationship between SOCS3 and pSTAT3, a panel of 9 pancreatic cancer cell lines were analyzed; we also observed highly activated STAT3 and lower expression of SOCS3 in most cell lines (Fig. 1d , Additional file 1: Figure S1B), suggesting that SOCS3 expression might be negatively correlated with that of pSTAT3 in PDAC.

**Fig. 1:** Expression of pSTAT3 and SOCS3 in PDAC and matched pericancerous tissue. **a** The representative images of immunohistochemistry staining of IL-6, pSTAT3, DNMT1, DNMT3a and SOCS3 in one matched PDAC (T) and pericancerous tissue (P) (20 × objective). **b** Statistical analysis of the IHC scores for the expression of IL-6, pSTAT3, DNMT1, DNMT3a and SOCS3 in the five pairs of PDAC and pericancerous tissue. **c** Protein expression levels of pSTAT3, STAT3 and SOCS3 were examined in five pairs of PDACs (T) and their matched pericancerous tissues (P) using western blots. **d** Protein expression levels of pSTAT3, STAT3 and SOCS3 were analyzed in nine pancreatic cancer cell lines using western blots

### IL-6/STAT3 signaling activation increased expression of DNMT1 and negatively regulated SOCS3 expression

As noted above, SOCS3 was downregulated and STAT3 was activated in pancreatic cancers. We next used real-time PCR and western blots to confirm the correlation between STAT3 activity and SOCS3 expression in pancreatic cancer cell lines. According to our studies, Aspc1 and Panc1 cells had relatively lower expression of pSTAT3 while Bxpc3 and Capan2 cells had relatively higher expression of pSTAT3. We thus selected them as our cell models. IL-6 and S31-201 are agonist and inhibitor of the IL-6/Jak-2/STAT3 signaling pathway, respectively. Panc1 cell proliferation increased by treatment with IL-6 and Bxpc3 cell proliferation was inhibited by treatment with S31-201 (Additional file 1: Figure S1C). As shown in Figs. 2a and b, IL-6 treatment reduced SOCS3 levels and activated STAT3 in Aspc1 and Panc1 cells. Conversely, S3I-201 treatment in Bxpc3 and Capan2 cells increased SOCS3 mRNA and protein levels. This phenomenon revealed that SOCS3 expression was negatively regulated by pSTAT3. However, SOCS3 was conventionally induced by IL-6 signaling [32–35]. Because previous studies found that IL-6 could induce DNMT1 expression, we took the methylation modification of the SOCS3 gene into consideration. To study whether IL-6 could induce DNA hypermethylation in PDAC, we evaluated the expression of two representative DNMTs, DNMT1 and DNMT3a, in Aspc1and Panc1 cell lines with IL-6 stimulation. Substantial increases in pSTAT3 and DNMT1 expression were observed in both cells but DNMT3A expression was not substantially increased. Therefore, the results suggest that IL-6 increased DNA methylation mainly through up-regulation of DNMT1. We further found that S3I-201 treatment could decrease the level of DNMT1 expression, but not DNMT3A expression, in Bxpc3 and Capan2 cell lines (Fig. 2c). These data indicate that in pancreatic cancer cells, IL-6 upregulated DNMT1 by activating the IL-6/STAT3 signaling pathway.

**Fig. 2:** IL-6/STAT3 signaling activation increased expression of DNMT1 and negatively regulated SOCS3 expression. **a** Protein expression levels of pSTAT3 and SOCS3 were analyzed in Aspc1 and Panc1 cells after IL-6 (100 ng/ml) and Bxpc3 and Capan2 cells after S31-201 (a STAT3 inhibitor, 10μM) treatment for 24 h using western blots. **b** mRNA expression levels of SOCS3 were analyzed in Aspc1 and Panc1 cells after IL-6 (100 ng/ml) and Bxpc3 and Capan2 cells after S31-201 (a STAT3 inhibitor, 10μM) treatment for 24 h using quantitative real-time PCR. Results were expressed as SOCS3/ACTIN. Gene expression measurements were performed in triplicate. Bars represented the mean ± SD. * *p* < 0.05, ** *p* < 0.01. **c** Protein expression levels of pSTAT3, STAT3, DNMT1 and DNMT3a were analyzed in Aspc1 and Panc1 cells after IL-6 (100 ng/ml) and Bxpc3 and Capan2 cells after S31-201 (a STAT3 inhibitor, 10μM) treatment for 24 h using western blots

### STAT3 represses SOCS3 expression through recruitment of DNMT1 in pancreatic cancer

Because we found that IL-6 could upregulate DNMT1 while downregulate SOCS3 levels in pancreatic cancer cell lines, we further analyzed the possible correlation between IL-6 induced DNMT1 expression and methylation modification of SOCS3. We used MSP to analyze the methylation status of the promoter regions of SOCS3 near the recognized STAT3-SOCS3 binding sites in pancreatic cancer cell lines. The structure of SOCS3 and the location of the CpG islands are shown in Fig. 3a. We found a negative correlation between promoter methylation and basal SOCS3 protein levels shown in Fig. 1 (Fig. 3b). As shown in Fig. 3c, the methylation level of SOCS3 gene in Aspc1 and Panc1 cells increased after IL-6 incubation for 24 h. In contrast, STAT3 inhibitor (S3I-201) treatment for 24 h could eliminate the methylation level of the SOCS3 gene in Bxpc3 and Capan2 cells. Thus, we could conclude that IL-6/STAT3 signaling might influence the methylation level of the SOCS3 gene.

**Fig. 3:** STAT3 represses SOCS3 expression through recruitment of DNMT1 in pancreatic cancer. **a** Structure of the SOCS3 gene. Bottom line is a genomic sequence of SOCS3 gene containing Exon 1, Intron 1, and Exon 2. The translation start site ATG is defined as +1. The grey vertical bar represents the recognized STAT3-SOCS3 binding site (−1046 through −1038). The arrows indicate primers used for MSP. **b** The SOCS3 gene promoter methylation status was analyzed in four pancreatic cancer cell lines using MSP. M and U, PCR products of methylated and unmethylated alleles, 155bp and 158bp, respectively; Con(M), methylation positive control; Con(U), positive control for unmethylation. **c** The SOCS3 gene promoter methylation status was analyzed in Aspc1 and Panc1 cells after IL-6 (100 ng/ml) and Bxpc3 and Capan2 cells after S31-201 (a STAT3 inhibitor, 10μM) treatment for 24 h using MSP. **d** Bxpc3 cells were infected with lentiviral vectors carrying control vector (EV) or DNMT1-specific shRNAs (shDNMT1), then followed by puromycin selection. Protein expression levels of DNMT1 and SOCS3 were analyzed in Bxpc3/EV and Bxpc3/shDNMT1 cells in the absence or presence of IL-6 (100 ng/ml) for 24 h. **e** Protein expression levels of SOCS3 were analyzed in Bxpc3 cells after 5-Aza (5μM) treatment for 72 h (with medium changed every day). Protein expression levels of SOCS3 were also analyzed in Panc1 cells which were cultured in the presence of IL-6 (100 ng/ml) or 5-Aza (5μM) 72 h (with medium changed every day) using western blots. **f** Panc1 cells were co-transfected with the indicated plasmids (reporter plasmid EV alone or DNMT1 plasmid simultaneously). Then, 24 h after the transfection, the cells were treated with IL-6 (100 ng/ml) or 5-AZA (5μM) for 48 h, and the luciferase activity was measured. **g** Lysates of Bxpc3 cells were subjected to immunoprecipitation with rabbit IgG or pSTAT3 antibody, and then followed by western blot to detect the interaction of phosphorylated STAT3 with DNMT1. The effect of IL-6 on the interaction between phosphorylated STAT3 and DNMT1 in Panc1 cells were also analysed using western blots. * represents the location of DNMT1 (183 kd)

In order to confirm our postulation, we further silenced DNMT1 and analyzed SOCS3 expression in the presence of IL-6. We found that SOCS3 expression was dramatically increased and could be enhanced by IL-6 treatment in Bxpc3 cells with shRNA knockdown of DNMT1 (Fig. 3d). To further confirm that SOCS3 expression loss was caused by promoter methylation, we incubated Bxpc3 cells with 5-AZA, an inhibitor of DNA methylation and this treatment could significantly upregulate SOCS3 expression. Similar western blot analyses showed that in the presence of 5-AZA, IL-6 mediated down-regulation of SOCS3 in Panc1 cells was reversed (Fig. 3e). In conclusion, these data suggest that the IL-6/STAT3 signaling pathway downregulated SOCS3 expression by inducing DNMT1 mediated gene methylation.

To observe the effect of pSTAT3 and DNMT1 on SOCS3 promoter activity, we next transfected Panc1 cells with a reporter vector encoding Luciferase under control of the SOCS3 promoter (PGL3-SOCS3). Concurrent IL-6 treatment or DNMT1 plasmid transfection with the SOCS3 reporter construct decreased SOCS3 promoter activity. Nevertheless, IL-6 and 5-AZA treatment simultaneously could abolish pSTAT3-mediated repression of SOCS3 transcription (Fig. 3f). We could conclude from the above results that there must be some association among activated STAT3, DNMT1 and SOCS3. Therefore, we examined whether STAT3 could form complexes with DNMT1 in pancreatic cancer cells using co-immunoprecipitation assay.

We observed that endogenous pSTAT3 did interact with DNMT1 in Bxpc3 cells and IL-6 treatment enhanced the interaction in Panc1 cells (Fig. 3g). So we considered that pSTAT3 repressed SOCS3 expression through increasing DNMT1 expression and recruiting DNMT1 to the promoter region of SOCS3 in pancreatic cancer according to our studies.

### SOCS3 induces pancreatic cancer cell apoptosis and cell cycle arrest

Our results suggest a probable mechanism of decreased expression of SOCS3 in PDAC. To further elucidate the role of SOCS3 during pancreatic cancer development, we selected Bxpc3 and Panc1 cells which had relatively low and high expression of SOCS3 as our cell models. Protein level of SOCS3 was effectively enhanced after transfection with expression vector in Bxpc3, and SOCS3 knockdown in Panc1 was efficient after transfection with siSOCS3 1# compared to siNC. (Fig. 4a). The CCK8 assay showed that overexpression of SOCS3 could remarkably inhibit Bxpc3 cell growth (Fig. 4b). We next examined cell cycle and apoptosis using flow cytometry. Analysis of apoptosis using Annexin V and PI staining revealed that overexpression of SOCS3 increased apoptosis, whereas silencing SOCS3 decreased apoptosis (Fig. 4c, e). Cell cycle was blocked mainly at the G1-S transition by SOCS3 according to our studies (Fig. 4d, e). Consistent with these results, the western blot data showed that cell cycle-related protein CYCLIND1 and anti-apoptotic protein BCL-2 were downregulated in Bxpc3/SOCS3 OE cells, and upregulated in Panc1/ siSOCS3 cells (Fig. 4f). The results shown in Fig. 4f also suggest that downregulation of SOCS3 effectively enhanced the expression level of activated pSTAT3 and its downstream target genes CYCLIND1 and BCL-2.

**Fig. 4:** SOCS3 induces pancreatic cancer cell apoptosis and cell cycle inhibition. **a** Protein level of SOCS3 was effectively enhanced after transfection with expression vector in Bxpc3, and SOCS3 knockdown in Panc1 was efficient after transfection with siSOCS3 1# compared to siNC. **b** The CCK8 assay was used to examine cell growth of SOCS3 gene stably transfected Bxpc3 cells and a reduction of absorbance was observed at 24 h, 48 h and 72 h (*P* < 0.01). **c** Panc1 and Bxpc3 cells were transiently transfected with SOCS3 siRNA and SOCS3 expression vector, respectively. Cell apoptosis was measured using the flow cytometry 48 h post transfection. **d** The cell cycle distribution of SOCS3-modulated Panc1 and Bxpc3 cells was analyzed using the flow cytometry. **e** The proportions of apoptosis cells and cells in different phases of cell cycle were quantified. Data represents three independent experiments in triplicate. **f** Protein expression levels of cell apoptosis and cell cycle related genes were analyzed in Bxpc3 and Panc1 cells 48 h after transfection using western blots

### SOCS3 inhibits migration and invasion of pancreatic cancer cells in vitro

To further evaluate the role of SOCS3 in the metastasis of pancreatic cancer cells, we used wound healing and transwell invasion assays. The results showed that within 24 h, Panc1 cells transfected with siRNA against SOCS3 occupied approximately 77 % of the wound, while Panc1 cells with control siRNA covered approximately 64 % of the wound, indicating that knockdown of SOCS3 promoted the migration of Panc1 cells. Similarly, transwell assays showed that more Panc1 cells migrated through the matrix gel when SOCS3 expression was inhibited (Fig. 5a, b, c). A gain-of-function assay was also conducted by transfecting SOCS3 cDNA plasmid into Bxpc3 cells. As expected, overexpression of SOCS3 suppressed the migration and invasion capability of Bxpc3 cells (Fig. 5a, b, c). And we performed western blotting on invasion related proteins. The results showed a notably elevated protein level of MMP-2 and MMP-9 for Panc1/ siSOCS3 cells as compared with control cells (Fig. 5d). Conversely, the expression levels of MMP-2 and MMP-9 were reduced in Bxpc3/SOCS3 OE cells. Taken together, these results softened our statement regarding the inhibition of SOCS3 in migration and invasion of pancreatic cancer cells.

**Fig. 5:** SOCS3 inhibits migration and invasion of pancreatic cancer cells in vitro. **a** The wound healing migration assays were carried out in Panc1 cells after transfection with siSOCS3 as well as Bxpc3 cells after transfection with overexpression vector of SOCS3. Microscopic observations were recorded at 0, 8 and 24 h after scratching the cell surface (100×). Representative images from every independent experiment were shown. **b** Transwell invasion assay with matragel were performed in Panc1/siSOCS3 and Bxpc3/ SOCS3 OE cells (100×). **c** Quantitative analysis of the wound closure rates and invasion cells. The percentage of the wound healing was calculated as (the width of wound at 0 h - the width of wound at 24 h)/ the width of wound at 0 h. All experiments were carried out in triplicate. **d** Protein expression levels of MMP-2 and MMP-9 were analyzed in Bxpc3 and Panc1 cells 48 h after transfection using western blots

### Overexpression of SOCS3 suppresses tumor formation in vivo

To determine whether SOCS3 was involved in pancreatic cancer tumourigenesis, equal numbers (1 × 10^7^) of Bxpc3 cells transfected with stable SOCS3 gene overexpression or control vector were subcutaneously injected into nude mice. Six weeks after injection of the cells, mice were sacrificed and the volume and weight of the tumors were recorded. As shown in Fig. 6a and b, the overexpression of SOCS3 decreased the size and weight of the xenograft local tumor compared with control vector groups.

**Fig. 6:** Nude mice tumor formation assay and the expression of SOCS3 in the tissue microarray. **a** Images of xenograft tumors in nude mice formed by SOCS3 gene stably transfected Bxpc3 cells and the controls. **b** Tumor volume and weight of xenograft tumors in nude mice were quantitatively evaluated. **c **Represenative staining patterns of negative IHC staining of SOCS3 in pancreatic cancer tissue sample (T1) while moderate staining in matched pericancerous tissue (P1) in the tissue microarray. The image P2 was classified as weak staining of SOCS3 in the pericancerous tissue. **d** Quantification of SOCS3 IHC staining in the pancreatic cancer tissue microarray (The difference between pancreatic cancer and pericancerous tissues is significant, *P* = 0.005). **e** Kaplan-Meier survival method and log-rank test were used to evaluate overall survival and compare the differences between the two groups based on the SOCS3 status, *P* = 0.034

### Association between SOCS3 expression and clinicopathological parameters in PDAC

A tissue microarray that included pancreatic cancers (*n* = 90) and matched pericancerous tissues was used for the immunohistochemistry analysis of SOCS3 protein expression.

Figure 6c shows representative positive and negative staining images of SOCS3. We found that nearly 80 % of the pericancerous tissues had positive SOCS3 staining (16.7 % with moderate staining and 63.3 % with weak staining), whereas only 63.3 % of the tumors had positive SOCS3 staining (7.8 % with moderate staining and 55.5 % with weak staining) (Fig. 6d). The difference in SOCS3 protein expression between pericancerous and cancer tissues was statistically significant (*p* = 0.005). The association of SOCS3 expression with the clinicopathological variables of pancreatic cancer patients was shown in Table 2. Low SOCS3 expression was associated with larger tumor volume (*p* = 0.037), lymph node metastasis (*p* = 0.038) and advanced TNM stage (*p* = 0.001), but not with other clinical parameters. The median survival after operation was 24 and 42 months for negative and positive SOCS3 expression, respectively. Kaplan-Meier survival curve showed that the overall survival rate was significantly lower in patients with negative SOCS3 expression (Fig. 6e). Furthermore, multivariate analysis through the Cox proportional hazard model was conducted to determine the independent prognostic factor. We observed that low expression of SOCS3 and pN1 in tumors was associated with a poor prognosis independent of other clinical covariates, and the pTNM stage I was associated with a better prognosis compared to pTNM stage IIB (Table 3).

**Table 3:** Univariate and multivariate analysis of different prognostic parameters in 90 pancreatic cancer patients after pancreaticoduodenectomy

Parameters	Category	No.	Univariate		Multivariate	
			3-year OS (%)	*p*	RR (95 % CI)	*P*
Age				0.664		
	<60	41	34.1			
	≥60	49	34.7			
Sex				0.053		
	Male	57	26.3			
	Female	33	48.5			
Tumor Volume(cm3)				0.472		
	≤50	57	30.4			
	>50	33	41.2			
pT stage				0.775		
	T1	5	20.0			
	T2	70	35.7			
	T3	15	33.3			
pN stage				0.047		
	N0	51	43.1		1	
	N1	39	23.1		6.539 (1.266 to 33.764)	0.025
pTNM stage				0.033		
	I	40	47.5		0.079 (0.015 to 0.423)	0.003
	IIA	9	33.3			
	IIB	41	22		1	
SOCS3 expression				0.034		
	negative	33	24.2		1.815 (1.037 to 3.179)	0.037
	positive	57	40.4		1	

## Discussion

A link between chronic inflammation and cancer risk has been established [36, 37]. The IL-6/STAT3 signaling axis is recognized as a mechanistic link between the inflammatory tumor microenvironment and pancreatic cancer [38, 39], which promotes tumor initiation and progression not only through the regulation of oncogenes [40], but also by epigenetic modification of tumor suppressor genes [41].

However, the mechanism of the persistent aberrant activation of this signaling pathway in PDAC remains unclear. In the present study, we found for the first time that IL-6/STAT3- mediated SOCS3 gene methylation via DNMT1 may account for the imbalance of this signaling pathway. We also identified SOCS3 as a tumor suppressor gene important for pancreatic tumor growth and metastasis.

As a key negative feedback regulator of the IL-6/STAT3 signaling pathway, SOCS3 expression is usually induced upon IL-6 stimulation via Janus kinas 2 (JAK-2) /STAT3 under physiological conditions [15, 42]. In contrast, we demonstrated that SOCS3 expression was down-regulated in PDAC tissues while pSTAT3 expression was up-regulated. And SOCS3 induction was decreased in response to IL-6 in pancreatic cancer cells in our study. To illustrate the contradiction, the epigenetic modification was taken into consideration. Some inflammatory factors were reported to change the methylation status of the SOCS3 promoter and further inhibit SOCS3 expression [43, 44], but the mechanisms were not clear enough. We showed that DNMT1 other than DNMT3a, a conventional DNA methylation inducer, could be upregulated by IL-6/STAT3 signaling. This finding is in agreement with previous reports [45–47]. It was also reported that SOCS3 expression in ulcerative colitis-related colorectal cancer was effectively regulated by IL-6 via DNMT1 [48]. Our study further showed that demethylation treatment or DNMT1 knocked down could reverse IL-6 mediated down-regulation of SOCS3 in pancreatic cancer cells. Therefore, we proposed that SOCS3 epigenetic silence was due to IL-6/STAT3 signaling pathway induced methylation via increased DNMT1.

Although pSTAT3 seems to act mainly as a transcription activator, transcriptional repression by pSTAT3 through interacting with NF-κB [43], c-jun [49], HDAC1 [50] and DNMT1 [51] has also been described. This report provides the evidence that oncogenic STAT3 promotes epigenetic gene silencing in synergy with DNMT1. Binding of pSTAT3 to a gene promoter, as demonstrated here for SOCS3, could be the step that provides an anchor for DNMT1 that directly mediates DNA methylation in pancreatic cancer.

There have been varying findings concerning the roles of SOCS3 in tumourigenesis and tumor progression. The association of SOCS3 expression with the biological behavior of pancreatic cancer cells and clinico-pathological features in human PDAC has not been investigated. Our study first demonstrated that SOCS3 expression was down-regulated in PDAC tissues and overexpression of SOCS3 decreased the proliferation and invasion potential of pancreatic cancer cells both in vivo and vitro. Furthermore, in our microarray analysis, we found that low expression of SOCS3 was a significant predictor for larger tumor volume, lymph node metastasis, advanced TNM stage and even poorer overall survival in PDAC patients. This is similar to the role of SOCS3 in lymphoma [52], prostate cancer [53] and hepatocellular cancer [54]. Therefore, we conclude that SOCS3 is a candidate tumor suppressor-gene of PDAC.

The limitation of the study is the up-regulation of pSTAT3 or down-regulation of SOCS3 is not an universal feature of various cancer cell lines, which might result from the heterogeneity of different cancer cell lines. Besides, cell biological behavior depends on multiple signaling pathways. For Aspc1 and Panc1 cells, although the STAT3 signaling pathway might not be the main pathway which plays a decisive role in their biological behavior in vitro, they are greatly influenced by the inflammatory microenvironment in vivo. In the present study, we treated Aspc1 and Panc1 cells which had endogenous relatively low expression of pSTAT3 with IL-6 in vitro, to partially recapitulate the inflammatory microenvironments in vivo. Their malignant biological behaviors enhanced, as previously reported when IL-6/STAT3 signaling is activated [55, 56]. Although SOCS3 levels in Aspc1 and Panc1 cells are relatively high compared to others in vitro, we found a significantly reduced expression of SOCS3 after treatment with IL-6.

Another discrepancy is the inconsistency between the expression level of SOCS3 protein and the differentiated degree of pancreatic cancer cell lines. As reported in numerous publications, cancer progression is a multistep process that requires involvement of several biological mechanisms and sequential acquisition of multiple genetic lesions. Therefore, we presume that SOCS3 may cooperate with other genes to ultimately determine cancer biological behaviors. This would explain why there might be a fraction of tumors positive to SOCS3 but with poorly differentiated characteristics (i.e.Panc1 cells). What is clear from our data is that Panc1 cells acquire more aggressive features when SOCS3 is knocked down, which is in accordance with other previously published studies. Moreover, we provide evidences that cell proliferation and invasion related proteins change, which highlight again a relevant role of SOCS3 in tumor aggressiveness. Nevertheless, further study about this issue needs to be done in our future work.

## Conclusions

In summary, our results indicate that activated IL-6/STAT3 signaling could induce SOCS3 methylation via DNMT1 in pancreatic cancers, which may account for the imbalance of the signalling pathway. We also identify SOCS3 as a tumour suppressor gene important for pancreatic tumour growth and metastasis. Ultimately, these data suggests that various inhibitors of STAT3 or DNMT1 may become novel strategies for treating pancreatic cancer.

## Additional file

Additional file 1: Figure S1. (A) Normalized band quantization data of pSTAT3 and SOCS3 in Fig. 1c by Image J between matched pancreatic cancer and pericancerous tissues were used to confirm our claim. (B) Normalized band quantization data of pSTAT3 and SOCS3 in Fig. 1d by Image J were evaluated. (C) The CCK8 assay was used to evaluate the proliferation of Panc1 cells after treatment with IL-6 (100 ng/ml) at 0 h, 24 h and 48 h. After seeding Bxpc3 cells for 24 h, we treated Bxpc3 cells with S31-201 (10μM). The CCK8 assay was used to evaluate the proliferation of Bxpc3 cells after treatment with S31-201 at 0 h, 24 h and 48 h. (JPG 973 kb)

## Abbreviations

IL-6: Interleukin-6
STAT3: Signal transducer and activator of transcription 3
SOCS3: Suppressor of cytokine signaling 3
DNMT1: DNA Methyltransferase 1
pSTAT3: phosphorylated STAT3
PDAC: Pancreatic ductal adenocarcinoma
JAK-2: Janus kinase 2
5-AZA: 5-aza-2-deoxycytidine
qRT-PCR: Quantitative reverse transcription-polymerase chain reaction
MSP: Methylation-specific PCR
OS: Overall survival
